RETRACTED

# Over-Expression of Superoxide Dismutase Ameliorates Cr(VI) Induced Adverse Effects via Modulating Cellular Immune System of *Drosophila melanogaster*

**DOI:** 10.1371/journal.pone.0088181

**Published:** 2014-02-04

**Authors:** Prakash Pragya, Arvind Kumar Shukla, Ramesh Chandra Murthy, Malik Zainul Abdin, Debapratim Kar Chowdhuri

**Affiliations:** 1 Embryotoxicology Section, CSIR-Indian Institute of Toxicology Research, Lucknow, Uttar Pradesh, India; 2 Analytical Section, CSIR-Indian Institute of Toxicology Research, Lucknow, Uttar Pradesh, India; 3 Department of Biotechnology, Jamia Hamdard, New Delhi, India; CSIR-Central Drug Research Institute, India

## Abstract

The evolutionarily conserved innate immune system plays critical role for maintaining the health of an organism. However, a number of environmental chemicals including metals are known to exert adverse effects on immune system. The present study assessed the *in vivo* effect of a major environmental chemical, Cr(VI), on cellular immune response using *Drosophila melanogaster* and subsequently the protective role of superoxide dismutase (SOD) based on the comparable performance of the tested anti-oxidant enzymes. The immuno-modulatory potential of Cr(VI) was demonstrated by observing a significant reduction in the total hemocyte count along with impaired phagocytic activity in exposed organism. Concurrently, a significant increase in the percentage of Annexin V-FITC positive cells, activation of DEVDase activity, generation of free radical species along with inhibition of anti-oxidant enzyme activities was observed in the hemocytes of exposed organism. In addition, we have shown that ONOO^−^ is primarily responsible for Cr(VI) induced adverse effects on *Drosophila* hemocytes along with O_2_^−^. While generation of O_2_^−^/ONOO^−^ in Cr(VI) exposed *Drosophila* hemocytes was found to be responsible for the suppression of *Drosophila* cellular immune response, Cr(VI) induced alteration was significantly reduced by the over-expression of *sod* in *Drosophila* hemocytes. Overall, our results suggest that manipulation of one of the anti-oxidant genes, *sod*, benefits the organism from Cr(VI) induced alteration in cellular immunity. Further, this study demonstrates the applicability of *D. melanogaster* to examine the possible effects of environmental chemicals on innate immunity which can be extrapolated to higher organisms due to evolutionary conservation of innate immune system between *Drosophila* and mammals.

## Introduction

The ever-increasing human needs have led to countless anthropogenic activities resulting in the release of thousands of chemicals into the environment. The consequence has been detrimental effects of these chemicals on the exposed organism [1]. Since immune system is the first line of defense mechanism in all metazoans, it is likely to be the primary target of environmental chemicals. Considering the importance of this system, there is growing concern to elucidate the effects of such chemicals on the immune system of exposed organism [2]. It has been reported that environmental chemical can impair the immune defense of an organism which eventually leads to chemical induced immunological disorders [3]. Among environmental chemicals, heavy metals have been reported to cause imbalance in the cellular immune homeostasis in exposed organism [4], [5].

RETRACTED

One of the heavy metals, chromium (Cr), has widespread environmental existence due to its extensive application in diverse industrial processes such as chrome plating, chrome pigmenting, leather tanning, steel manufacturing etc [6]. It exists in several oxidation states in the environment of which Cr(III) and Cr(VI) are the most stable and common forms having biological significance. Cr(III) is a macro-nutrient while Cr(VI), a Class I A human carcinogen [7], is the most toxic form of Cr due to its higher solubility in water, rapid permeability through biological membranes and subsequent interaction with intracellular proteins and nucleic acids [8]. Earlier studies revealed that Cr(VI) induced reactive oxygen species (ROS) generation causes oxidative stress in the exposed organism which can exert various adverse effects such as apoptosis, modulation of intracellular oxidized states, oxidative deterioration of macro-molecules among others [9], [10]. Although limited studies are available to show the immuno-suppressive potential of Cr(VI) in exposed organisms [11]–[13], those studies were essentially carried out either *in vitro* or in organisms which have both innate as well as adaptive immunity. Due to the presence of both types of immunity, immune system in those organisms becomes complex and therefore, molecular mechanism underlying the chemical induced modulation of primary innate immune defense remains to be elegantly evaluated.

Due to the association of Cr(VI) induced adverse effects with oxidative stress, different anti-oxidants including various modulators of ROS [superoxide dismutase (SOD), catalase] were shown to provide protection against Cr(VI) induced adversities in exposed organism [9], [14]. Thus, cytosolic enzyme Cu/Zn SOD, a key enzyme in the dismutation of superoxide radicals [15], assumes significance in the context of Cr(VI) induced adverse biological effects on the innate immune system of exposed organism.

In order to have insight into the mechanism of Cr(VI) induced alteration of cellular immunity and evaluation of possible immuno-protective role of SOD, a suitable model organism with well-characterised genetic network is preferred. In this context, fruit fly *Drosophila*, a well established model organism to study basic principles of innate immunity [16], has been chosen. It relies only on evolutionarily conserved multiple innate immune mechanisms for its defense. The innate immunity in *Drosophila* comprise cellular and humoral responses [17]. Cellular immune response in this organism is mediated by its hemocytes. These cells show extensive homology with vertebrate myeloid lineage especially with mammalian leukocytes [18] eventually protecting the organism from pathogenic infection. In addition, ease of genetic manipulation, limited ethical concern as well as recommendation from European Centre for the Validation of Alternative Methods (ECVAM) for toxicological research and testing makes this model useful to study immune response after chemical exposure [19].

RETRACTED

The present study, therefore, aims to examine Cr(VI) induced alterations of cellular immune response using *Drosophila* along with subsequent protection by over-expressing one of the major anti-oxidant genes, *sod*, in their hemocytes. Due to evolutionarily conserved innate immune response, the elucidation of Cr(VI) induced alterations in the cellular immunity of *Drosophila* would add to our understanding regarding innate immunity that can be affected by environmental chemicals in higher organisms.

## Materials and Methods

### Fly stocks and genetics

Wild type *D. melanogaster* (Oregon R^+^), Gal4-UAS transgenic lines namely Hemese-Gal4 (*He-Gal4*), *UAS-Sod*, *UAS-Sod RNAi* and *hml^Δ^-Gal4 UAS-2xEGFP* (a driven strain having constitutive expression of GFP in hemocytes) were used for the study. Necessary genotypes were generated by standard genetic crosses. The fly strains and their larvae were reared on standard *Drosophila* food medium (consisting of agar-agar, maize powder, sugar, yeast, nepagin and propionic acid) at 24±1°C [20]. Additional yeast supplement was provided for healthy growth of the organisms. All the chemicals of highest purity were obtained from Sigma, St Louis, MO, USA unless stated otherwise.

### Exposure schedule

Analytical grade Potassium dichromate (K_2_Cr_2_O_7_) (HiMedia Laboratories Ltd, Mumbai, India) and Sodium molybdate (Na_2_MoO_4_.2H_2_O) (Merck India Ltd, Mumbai, India) were used for the present study. In a recently conducted study, level of Cr(VI) in ground-water in the vicinity of industrial areas of a major city of Uttar Pradesh, India inhabited by humans was determined as ∼20.0 µg/ml [21]. We used three different concentrations of Cr(VI) (5.0, 10.0 and 20.0 µg/ml) that have environmental [22] and biological [23] relevance. Larvae of both control and exposed groups were grown on standard *Drosophila* food contaminated with or without the metal salt for 24 and 48 h. For Mo(VI) [another metal of the same group VI of periodic table and was used as a control], its 20.0 µg/ml concentration and 48 h exposure period were chosen. Control group received standard *Drosophila* food. All the experiments were carried out thrice with three independent biological replicates.

RETRACTED

### Quantitative estimation of metal level in the hemocytes of exposed organism

For detecting Cr levels in the larval hemocytes of different strains, approximately 3000 larvae each from control and exposed groups were taken. Hemocytes were isolated in phosphate-buffered saline (PBS) and the amount of Cr present in these cells was estimated using a flame and graphite furnace atomic absorption spectrophotometer (Flame & Graphite furnace AAS; ZEEnit 700; Analytik Jena AG, Germany). The data were presented as ng/ml.

### Immunofluorescence analysis and hemocyte imaging

Hemocytes were isolated from Drosophila larvae as described previously [18] with minor modifications. Briefly, the hemolymph having hemocyte population was suspended in Schneider's insect medium (SCM) supplemented with 10% fetal bovine serum (FBS; Invitrogen, USA) on a coverslip for adherence. The hemocytes were fixed in 4% paraformaldehyde (PFA) washed with PBS, permeabilized in 0.1% Triton-X 100 and then blocked with 0.1% bovine serum albumin (BSA).

Immunostaining of hemocytes was carried out by incubating the cells in hemocyte-specific Hemese (H2) antibody (1∶100 in 4% BSA) and cleaved caspase-3 antibody (1∶200 in 4% BSA; Cell Signaling, Danvers, MA, USA) overnight at 4°C followed by staining with Alexa-Fluor 488 goat anti-mouse (Invitrogen, USA) and Cy-3 conjugated goat anti-rabbit secondary antibodies respectively at 1∶200 dilutions in 4% BSA for 2 h. Nuclear staining was performed with 4′,6-diamidino-2-phenylindole (DAPI) (1 µg/ml in PBS). For microscopic examination, cells were mounted on a slide using Vectashield mounting medium (Vector Laboratories, Burlingame, CA). Immunofluorescence analysis was carried out by capturing the images on a Leica TCS SPE confocal microscope (Nussloch, Germany) and further processed using Adobe PhotoShop 7.0 software.

### Phagocytosis assay

The phagocytosis assay was carried out essentially by following a previously published method [24] with minor modifications. Briefly larval hemocyte suspension in SCM (supplemented with FBS) was incubated with E. coli-GFP, a Gram negative bacterium E.coli which is tagged with green fluorescent protein (GFP), at 25°C for 30 min. After incubation, cells were washed with PBS and 0.2% trypan blue was added to quench the non-phagocytosed bacteria. The number of hemocytes was normalized in control and Cr(VI) exposed groups and the phagocytic activity was determined according to the number of cells showing phagocytosis in each sample.

RETRACTED

### Flow cytometric analysis of larval hemocytes, apoptotic cell death and ROS level

Flow cytometry analysis was performed using a Becton Dickinson flowcytometer (BD Biosciences, New Jersey, USA). Ten thousand events were acquired per group and the data were analyzed using Cell Quest software (Mac OS 8.6).

The quantitative estimation of hemocytes isolated from hml^Δ^-Gal4 UAS-2xEGFP larvae was carried out. In brief, hemocytes were isolated in PBS and EGFP fluorescence was quantified at an excitation/emission wavelength of 495/519 nm.

For apoptotic cell death analysis, larval hemocytes were stained with Annexin V-FITC essentially following the manufacturer's protocol (Annexin V-FITC apoptosis detection kit). Briefly, cells were suspended in 500 µl of 1X binding buffer (media binding reagent) and subsequently Annexin V-FITC (5 µl) and propidium iodide (PI) (10 µl) were added to the cells. The cells were incubated at 24±1°C for 10 min in dark. The FITC signal was detected by FL1 (FITC detector) at 518 nm and Pl was detected by FL2 (phycoerythrin fluorescence detector) at 620 nm. The log of Annexin V-FITC and PI fluorescence was displayed on the X- and Y-axis of the data report respectively.

The levels of superoxide (O_2_^−^) and peroxide (H_2_O_2_) were measured in larval hemocytes using dihydroethidium (DHE; Invitrogen, USA) and 2′, 7′-dihydrofluorescein diacetate (H_2_DCFDA) respectively following the methods reported earlier [9], [25] with minor modifications. Briefly, isolated hemocytes were incubated with respective dyes at the final concentration of 10 µM for 1 h in dark at 24±1°C. Following a brief washing with PBS, cells were finally re-suspended in PBS for analysis. The fluorescence intensity of the oxidized derivatives of two dyes viz., 2-hydroxyethidium for DHE and 2′, 7′-dichlorofluorescein (DCF) for H_2_DCFDA was quantified at an excitation/emission wavelength of 535/617 nm and 492/517 nm respectively. The mean fluorescence intensity was used for the estimation of intracellular ROS level in each sample.

### Measurement of peroxynitrite (ONOO^−^) generation

Generation of peroxynitrite anion (ONOO^−^) in the cellular system was detected by peroxynitrite mediated oxidation of dihydrorhodamine 123 (DHR 123; Cayman Chemical, USA) to its fluorescent product rhodamine following a published method [26] with minor modifications. Briefly, hemocytes were incubated with 20 µM DHR 123 in PBS for 10 min at 24±1°C and fluorescence intensity of the dye was measured at an excitation/emission wavelength of 500/536 nm on a Varioskan Flash spectrofluorometer (Thermo Fisher Scientific, Finland). The generation of ONOO**^−^** was estimated by mean fluorescence intensity of the samples.

RETRACTED

### Biochemical assays for oxidative stress parameters and DEVDase activity

The absorbance of the coloured products in the following biochemical assays was measured on a Cintra 20 ultraviolet spectrophotometer (GBC Scientific Equipment, Melbourne, Australia).

Different oxidative stress parameters viz., SOD, catalase, thioredoxin reductase (TrxR) enzyme activities, m*alonyldialdehyde* content and total anti-oxidant capacity were measured in the larval hemocytes.

SOD (superoxide: superoxide oxidoreductase EC 1.15.1.1) enzyme activity in Drosophila hemocyte homogenate was measured following a published method [27] with minor modifications. Briefly, the assay reaction mixture consists of hemocyte sample (Fig. S1), cytochrome C, xanthine and xanthine oxidase in 3 ml potassium phosphate buffer containing EDTA at 25°C. One unit of enzyme activity is defined as the enzyme concentration required for inhibiting the rate of reduction of cytochrome C (optical density at 550 nm) by 50% under assay condition and results were expressed as specific activity in units/mg protein.

Catalase (CAT) (H_2_O_2_: H_2_O_2_ oxidoreductase EC 1.11.1.6) activity was measured by following its ability to split H_2_O_2_ within 1 min of incubation time. The reaction was then stopped by adding dichromate/acetic acid reagent and the remaining H_2_O_2_ was determined by measuring chromic acetate at 570 nm which is formed by reduction of dichromate/acetic acid in the presence of H_2_O_2_ as described earlier [28]. The results were expressed as µmoles H_2_O_2_/min/mg protein.

The activity of thioredoxin reductase (TrxR), a substitute for Drosophila glutathione reductase (GR) [29], was measured following a published method [30] with minor modifications. Briefly, to hemocyte homogenate, potassium phosphate and ethylenediaminetetraacetic acid (EDTA) (pH 7.4) were added. After an oxidation step in the presence of reduced nicotinamide adenine dinucleotide (NADPH) and 5,5-dithiobis (2-nitrobenzoate) (DTNB), TrxR activity in the sample was assessed at an absorbance of 412 nm. The results were expressed as nmoles NADPH oxidized/min/mg protein using molar extinction coefficient of 13.6 mM^−1^ cm^−1^.

The level of malondialdehyde (MDA) as a marker of lipid peroxidation (LPO) was determined based on the reaction with thiobarbituric acid (TBA) as reported earlier [31]. The assay mixture consisted of hemocyte homogenate, distilled water, 10% sodium do-decylsulphate (SDS) and 20% acetic acid solution (pH 3.5). Absorbance was measured at 532 nm against n-butanol and results were expressed as nmoles MDA formed/mg protein.

RETRACTED

Protein content in different samples was estimated essentially following a method reported earlier [32] using BSA as the standard.

Total anti-oxidant capacity (TAC) was estimated in the larval hemocytes following the method reported earlier [33] with minor modifications. In brief, hemocyte homogenate was added to diluted *2,2′-azino-bis-(3-ethylbenzothiazoline-6-sulphonic acid)* (ABTS) solution at 30°C (Fig. S2). The absorbance was measured at 734 nm exactly 1 min after initial mixing. The percentage inhibition of absorbance at 734 nm was calculated using trolox as an anti-oxidant standard.

DEVDase activity was measured in the larval hemocytes using caspase-3 colorimetric assay kit according to the manufacturer's protocol. In brief, hemocyte homogenate was mixed with 1X assay buffer and caspase-3 substrate and then the reaction mixture was incubated at 37°C for 1.5 h. Spectrophotometric detection of the chromophore p-Nitroaniline (pNA) at 405 nm was measured for caspase activity which was calculated in terms of µmol pNA released/min/ml of cell lysate.

### Determination of SOD activity by in-gel activity assay

The in-gel SOD activity assay was performed essentially following the method described previously [34] with minor modifications based on the reduction of nitroblue tetrazolium (NBT) by O_2_ **^−^** radical into a blue precipitate in the native poly-acrylamide gel. Briefly, hemocyte homogenate was loaded on a native poly-acrylamide gel and electrophoresed at 4°C for 3 h at 40 mA. Post electrophoresis, the gel was stained with SOD native gel stain comprising NBT, tetramethylethylenediamine (TEMED) and riboflavin in dark. Under fluorescent light, the achromatic bands (clear area) visualized on the gel indicate the SOD enzyme activity present in the sample.

### Measurement of the resistance of *Drosophila* larvae following bacterial infection

The survival of *Drosophila* larvae was measured after they were infected with a Gram negative bacterium, *Erwinia carotovora carotovora* 15 (Ecc15; DSMZ, Germany) as described previously [35] with minor modifications. Briefly, larvae were fed on the mixture of crushed banana and concentrated bacterial pellet in 2∶1 ratio for 30 min. The whole mixture was then transferred to a vial containing standard food medium. After 30 min, the larvae were washed in water and transferred individually to an agar plate for scoring at 29°C.

RETRACTED

### Statistical analysis

Prior to analysis, homogeneity of variance and normality assumption concerning the data was tested. Statistical significance of the mean values of different parameters was monitored in control and exposed groups using one way and two way analysis of variance (ANOVA). All the analysis in the same strain with the concentration of metal as a variable was done by one way ANOVA following Dunnett's test, while comparative analysis between different strains was performed using two way ANOVA followed by Bonferroni's test for multiple comparisons. Survival analysis was performed using log-rank test. All the statistical analyses were carried out by Prism software (GraphPad version 5.0, San Diego, CA, USA) after setting the level of statistical significance at *p*<0.05.

## Results

### Detection of metal in the hemocytes of exposed *Drosophila* larvae

A concentration- and time-dependent increase in Cr level was detected in the hemocytes of exposed larvae of different strains (Table S1). A non-significant (*p*>0.05) deviation in Cr levels was observed in the transgenic strains in comparison to that detected in Oregon R^+^ larvae. The level of metal in unexposed control larvae was beyond the level of detectable limit.

### Reduction in total hemocyte count in Cr(VI) exposed Oregon R^+^ larvae

We observed a concentration- and time-dependent reduction in the total hemocyte count in exposed Oregon R^+^ larvae with a maximum reduction of ∼56% at 20.0 µg/ml Cr(VI) after 48 h (Fig. 1A, D). Similar to reduced hemocyte number, a significant down-regulation in the gene expression level of *hemese* was also observed in exposed organism (Fig. S3A). Further, reduction in total hemocyte count observed in the exposed *hml^Δ^-Gal4 UAS-2xEGFP* larvae (Fig. 1B–C) was found to be comparable with Oregon R^+^.

**Figure 1:** Reduction of total hemocyte count (THC) in Cr(VI) exposed *D. melanogaster* larvae. Graphical representation of total hemocyte number (%) in Cr(VI) exposed Oregon R^+^ larvae after immunostaining by Hemese (H2) antibody (A). Hemocyte population in *hml^Δ^-Gal4 UAS-2xEGFP* larvae after Cr(VI) exposure (B). Graph representing total hemocyte count in Cr(VI) exposed *hml^Δ^-Gal4 UAS-2xEGFP* larvae as determined by flow cytometry (C). Data represent mean ± SD (n = 3) (20 larvae in each replicate). Significant differences were ascribed as *p<0.05; **p<0.01 and ***p<0.001 as compared to control. Representative confocal microscopic images of the hemocytes in control, 20.0 µg/ml Cr(VI) and 20.0 µg/ml Mo(VI) exposed Oregon R^+^ larvae for 48 h (D). Extreme right panel represents overlayed images of H2 (green) and DAPI (blue) stained cells. Scale bar: 20 µm.

RETRACTED

That the reduced total hemocyte count is indeed due to hexavalent Cr and not due to hexavalent form of another metal, was further confirmed by exposing the larvae to another metal Mo(VI). Unlike the above, we observed non-significant difference in the total hemocyte count in 20.0 µg/ml Mo(VI) exposed Oregon R^+^ larvae for 48 h in comparison to unexposed control (∼7% reduction; Fig. 1D).

### Inhibition of phagocytic activity in the hemocytes of Cr(VI) exposed organism

Earlier, it has been stated that the phagocytic activity of a cell can be attributed as an immunological biomarker [36] to demonstrate the potential of a chemical for immuno-modulation. In this context, we observed a significant inhibition of phagocytic activity in the hemocytes of Cr(VI) exposed organism (Fig. 2) with a maximum inhibition of ∼53% at 20.0 µg/ml after 48 h.

**Figure 2:** Inhibited phagocytic activity of the hemocytes of Cr(VI) exposed *Drosophila* larvae. Graph showing inhibition of phagocytic activity (%) in the hemocytes of Cr(VI) exposed Oregon R^+^ larvae. Bar graphs represent mean ± SD (n = 3) (10 larvae in each replicate). Statistical significance was *p<0.05; **p<0.01 and ***p<0.001 as compared to control.

### Increased apoptotic cell death in the hemocytes of Cr(VI) exposed organism

Since apoptosis can be the predominant mode of cell loss due to Cr(VI) exposure [37], we observed a concentration- and time-dependent increase in the % AV positive cells in Cr(VI) exposed Oregon R^+^ larvae with a maximum increase (∼31%) at 20.0 µg/ml of metal concentration after 48 h in comparison to control hemocyte population (Fig. 3A–B).

**Figure 3:** Increased apoptosis in the hemocyte population of Cr(VI) exposed Oregon R^+^ larvae. Quantitative graph of percent AV positive hemocytes in Cr(VI) exposed *Drosophila* larvae (A). Bar graphs represent mean ± SD (n = 3) (50 larvae in each replicate). Significance was ***p<0.001 in comparison to control. Representative dot plots for Annexin V-FITC and PI staining in the hemocytes of control (a) and 20.0 µg/ml Cr(VI) exposed (b) larvae for 48 h (B).

### Activation of DEVDase activity in the hemocytes of exposed Oregon R^+^ larvae

Similar to the detectable increase in AV positive hemocyte population in Cr(VI) exposed Oregon R^+^ larvae at higher concentrations of the test chemical, we also observed an increase in DEVDase (caspase 3-like) activity in the hemocytes of exposed organism. Maximum increase in DEVDase activity (∼360%) was observed in the hemocytes of larvae that were exposed to 20.0 µg/ml Cr(VI) for 48 h (Fig. 4A). Parallel to the DEVDase activity, immunofluorescence analysis using cleaved caspase-3 antibody also revealed activation of caspase-3 in the hemocytes of exposed organism (Fig. 4B).

RETRACTED

**Figure 4:** DEVDase (caspase 3-like) activity in the hemocytes of *Drosophila* larvae exposed to Cr(VI). Graphical representation of DEVDase activity (%) in the hemocytes of Oregon R^+^ larvae after their exposure to Cr(VI) (A). Data represent mean ± SD (n = 3) (50 larvae in each replicate). Significance in comparison to control was ascribed as *p<0.05; **p<0.01 and ***p<0.001. Representative confocal images of hemocytes from control and 20.0 µg/ml Cr(VI) exposed Oregon R^+^ larvae for 48 h (B). Extreme right panel represents overlayed images of H2 (green), DAPI (blue) and cleaved caspase-3 (red) antibody stained cells. Scale bar: 20 µm.

### Enhanced generation of O_2_^−^ in the hemocytes of Cr(VI) exposed Oregon R^+^ larvae

Concomitant with our observations on Cr(VI) induced reduction in total hemocyte count and apoptotic cell death, a significant increase in DHE and DCF fluorescence intensities in the hemocytes of Cr(VI) exposed Oregon R^+^ larvae with a maximum increase in DHE (∼302%; Fig. 5A) and DCF (∼267%; Fig. 5B) fluorescence at 20.0 µg/ml Cr(VI) after 48 h was observed as compared to control. Further, involvement of H_2_O_2_/OH was resolved by inhibiting the generation of OH radical in the hemocytes of 20.0 µg/ml Cr(VI) exposed *Drosophila* larvae after 24 and 48 h using N-acetylcysteine (NAC), which is reported to scavenge cellular H_2_O_2_ and OH radical [38]. We did not observe any significant beneficial effect on the total hemocyte count and apoptotic cell death of the hemocytes in larvae that were exposed to 10 mg/ml NAC and 20.0 µg/ml Cr(VI) together as compared to that observed with 20.0 µg/ml Cr(VI)-alone exposed organism (Fig. 6A–B; Fig. S4A). Non-significant alterations in the above parameters were observed after exposure of NAC alone to *Drosophila* larvae (data not shown).

**Figure 5:** Generation of free radicals in the hemocytes of *Drosophila* larvae exposed to Cr(VI). Graphs showing O_2_^−^ generation (A), H_2_O_2_ generation (B) and ONOO^−^ generation (C) in the hemocytes from control and Cr(VI) exposed Oregon R^+^ larvae. Values are mean ± SD (n = 3) (50 larvae in each replicate). Statistically significant differences were ascribed as *p<0.05; **p<0.01 and ***p<0.001 in comparison to control.

**Figure 6:** Effect of NAC, L-NAME, SNP on THC and apoptosis in *Drosophila* hemocytes after Cr(VI) exposure. Graphical representation of total hemocyte number (%) in 20.0 µg/ml of Cr(VI) exposed Oregon R^+^ larvae along with 10 mg/ml N-acetylcysteine (NAC) or 100 mM N-nitro-L-arginine methyl ester (L-NAME) or 50 µM sodium nitroprusside (SNP) after 24 and 48 h (A1). Representative confocal images of hemocytes from control, 20.0 µg/ml Cr(VI), 20.0 µg/ml Cr(VI) with 10 mg/ml NAC, 20.0 µg/ml Cr(VI) with 100 mM L-NAME and 20.0 µg/ml Cr(VI) with 50 µM SNP exposed Oregon R^+^ larvae after 48 h (A2). Scale bar: 20 µm. Twenty larvae were taken for each replicate. Graphical representation of percent AV positive hemocytes in *Drosophila* larvae exposed to 20.0 µg/ml Cr(VI) along with 10 mg/ml NAC or 100 mM L-NAME or 50 µM SNP for 24 and 48 h respectively (B1). Dot plots showing Annexin V-FITC and PI staining in the hemocytes of control (a), 20.0 µg/ml Cr(VI) (b), 20.0 µg/ml Cr(VI) with 10 mg/ml NAC (c), 20.0 µg/ml Cr(VI) with 100 mM L-NAME (d) and 20.0 µg/ml Cr(VI) with 50 µM SNP (e) exposed Oregon R^+^ larvae after 48 h (B2). Fifty larvae were taken for each replicate. Data represent mean ± SD (n = 3). Significant differences were ascribed as **p<0.01; ***p<0.001 in comparison to control and **^#^** *p*<0.05; **^##^** *p*<0.01 and **^###^** *p*<0.001 as compared to 20.0 µg/ml Cr(VI) exposure.

RETRACTED

### Peroxynitrite generation in the hemocytes of Cr(VI) exposed organism

A concentration- and time-dependent increase in DHR fluorescence was observed in the hemocytes of exposed organism with a maximum increase of ∼244% after 20.0 µg/ml Cr(VI) exposure for 48 h (Fig. 5C). On the other, inhibition of ONOO^−^ generation in the hemocytes of *Drosophila* larvae was achieved by exposing the organism to 100 mM N-nitro-L-arginine methyl ester [L-NAME; a nitric oxide synthase (NOS) inhibitor] [39] (Fig. S4B), along with Cr(VI) for 24 and 48 h. A significant increase in the total hemocyte count as well as decreased apoptotic cell death was observed in co-exposed larvae in comparison to that observed in 20.0 µg/ml Cr(VI)-alone exposed organism (Fig. 6A–B). When the larvae were exposed to 50 µM sodium nitroprusside [SNP; a potent nitric oxide (NO) generator] [40] (Fig. S4C) along with 20.0 µg/ml Cr(VI) for 24 and 48 h, we observed a significant reduction in the total hemocyte count and increased apoptotic cell death in the co-exposed group as compared to Cr(VI)-alone exposed group (Fig. 6A–B). However, exposure of L-NAME or SNP alone to *Drosophila* larvae non-significantly altered the above measured endpoints (data not shown).

### Generation of oxidative stress in the hemocytes of Cr(VI) exposed organism

A concentration- and time-dependent significant decrease in SOD activity in the hemocytes of Cr(VI) exposed larvae was observed [∼37% after 20.0 µg/ml Cr(VI) exposure for 48 h] (Fig. 7A). This observation was further confirmed by in-gel SOD activity assay which showed a trend similar to that observed by the biochemical assay (Fig. 7B). However, unlike SOD, we observed a significant decrease in CAT and TrxR activities only in the hemocytes of 20.0 µg/ml Cr(VI) exposed larvae (Fig. 7C–D). Concomitant with an inhibition of all the above tested enzyme activities, we observed a concentration- and time-dependent significant increase in MDA content in the hemocytes of exposed Oregon R^+^ larvae (Fig. 7E). Further, total anti-oxidant capacity (TAC) declined in a concentration- and time-dependent manner in the hemocytes of Cr(VI) exposed larvae with a maximum ∼45% decrease when the organism was exposed to 20.0 µg/ml Cr(VI) for 48 h (Fig. 7F).

RETRACTED

**Figure 7:** Generation of oxidative stress in the hemocytes of Cr(VI) exposed Oregon R^+^ larvae. Graphical representation of SOD activity in the hemocytes of control and Cr(VI) exposed *Drosophila* larvae by biochemical assay (A) and by in-gel activity assay after 48 h (B). Graphs depicting CAT activity (C), TrxR activity (D), MDA content (E) and total anti-oxidant capacity (TAC) (F) in the hemocytes of Cr(VI) exposed Oregon R^+^ larvae. Values are mean ± SD (n = 3) (Fifty larvae for each replicate). Significant differences were ascribed as *p<0.05; **p<0.01 and ***p<0.001 as compared to control.

### Decreased resistance of Cr(VI) exposed *Drosophila* after *Ecc*15 infection

We observed a concentration- and time-dependent decrease in the resistance (in terms of survival of larvae) of Cr(VI) exposed Oregon R^+^ larvae infected with *Ecc*15 in comparison to *Ecc*15 only infected organism [∼48% survival in 20.0 µg/ml Cr(VI) exposed larvae for 48 h following *Ecc*15 pathogenic infection] (Fig. 8). Before the resistance assay, bacterial load in infected larvae was ascertained by quantifying the bacterial level after natural infection (Fig. S5A).

**Figure 8:** Poor resistance of Cr(VI) exposed Oregon R^+^ larvae against *Ecc*15 infection. Survival (%) of *Drosophila* larvae that were exposed to Cr(VI) for 24 (A) and 48 (B) h followed by *Ecc*15 infection indicating resistance of an organism. Each survival curve in the graph represents mean survival of larvae from three independent experiments having 100 larvae in each and statistical significance was ascribed as **p<0.01 and ***p<0.001 as compared to control.

### Immuno-protective effect of *sod* against Cr(VI) induced alteration in cellular immunity

We observed a significant increase in the total hemocyte count in Cr(VI) exposed *He-Gal4>UAS-Sod* larvae [∼29% higher cell count after 20.0 µg/ml Cr(VI) exposure for 48 h] (Fig. 9A1–2; Fig. S3B) and less inhibition of phagocytic activity (∼23%) (Fig. 9B) as compared to the respective *He-Gal4* larvae. Further, significantly lesser number of AV positive cells were observed in exposed *He-Gal4>UAS-Sod* larvae (∼18%) as against that observed in *He-Gal4* larvae (∼32%) under similar experimental condition (Fig. 9C1–2). Concurrently, we observed ∼149% decreased DEVDase activity in the hemocytes of exposed *sod* over-expressed strain as compared to the respective *He-Gal4* larvae (Fig. 9D1–2). A similar trend for ROS (O_2_^.-^ and H_2_O_2_) (Fig. 9E1–2) and peroxynitrite (Fig. 9E3) generation, SOD and CAT (Fig. 9F1–2) activities, MDA content (Fig. 9F3), TrxR activity (Fig. 9F4) and TAC level (Fig. 9F5) was observed in the hemocytes isolated from the exposed larvae of *sod* over-expressing strain. Further, increased resistance of Cr(VI) exposed *He-Gal4>UAS-Sod* larvae was observed in comparison to the respective *He-Gal4* larvae after *Ecc*15 infection (Fig. 9G; Fig. S5B). When *sod* was genetically knocked down in the hemocytes of *Drosophila* (*He-Gal4>UAS-Sod RNAi*), we observed severe oxidative stress, increased apoptotic cell death of hemocytes along with similar exacerbating effect on other end-points in the said strain as compared to that seen in respective *He-Gal4* larvae (Fig. 9).

**Figure 9:** Protective effect of *sod* over-expression on *Drosophila* cellular immune response after Cr(VI) exposure. Comparative hemocyte population in *He-Gal4*, *UAS-Sod*, *He-Gal4>UAS-Sod*, *UAS-Sod RNAi* and *He-Gal4>UAS-Sod RNAi* larvae after 48 h Cr(VI) exposure (A1). Representative microscopic images of hemocytes from control and in 20.0 µg/ml Cr(VI) exposed larvae for 48 h (A2). Phagocytic activity (%) of hemocytes of *He-Gal4*, *UAS-Sod*, *He-Gal4>UAS-Sod*, *UAS-Sod RNAi* and *He-Gal4>UAS-Sod RNAi* larvae after 48 h Cr(VI) exposure (B). Percent AV positive hemocytes in 48 h Cr(VI) exposed *He-Gal4*, *UAS-Sod*, *He-Gal4>UAS-Sod*, *UAS-Sod RNAi* and *He-Gal4>UAS-Sod RNAi* larvae (C1). Representative dot plots for Annexin V-FITC and PI staining in the hemocytes from *He-Gal4* control (a) and 20.0 µg/ml Cr(VI) exposed *He-Gal4* (b), *UAS-Sod* (c), *He-Gal4>UAS-Sod* (d), *UAS-Sod RNAi* (e) and *He-Gal4>UAS-Sod RNAi* (f) larvae for 48 h (C2). Comparative DEVDase activity in the hemocytes of *He-Gal4*, *UAS-Sod*, *He-Gal4>UAS-Sod*, *UAS-Sod RNAi* and *He-Gal4>UAS-Sod RNAi* larvae exposed to Cr(VI) for 48 h (D1). Representative confocal images of hemocytes from control and 48 h, 20.0 µg/ml Cr(VI) exposed larvae (D2). Comparative levels of O_2_^.−^ (E1), H_2_O_2_ (E2) and ONOO^−^ (E3) generation in the hemocytes of 48 h Cr(VI) exposed *He-Gal4*, *UAS-Sod*, *He-Gal4>UAS-Sod*, *UAS-Sod RNAi* and *He-Gal4>UAS-Sod RNAi* larvae. Graphical representation of SOD activity (F1), CAT activity (F2), MDA content (F3), TrxR activitity (F4) and TAC (F5) in the hemocytes of *He-Gal4*, *UAS-Sod*, *He-Gal4>UAS-Sod*, *UAS-Sod RNAi* and *He-Gal4>UAS-Sod RNAi* larvae that were exposed to Cr(VI) for 48 h. Representation of the survival (%) of 20.0 µg/ml Cr(VI) exposed *Drosophila* larvae (*He-Gal4*, *UAS-Sod*, *He-Gal4>UAS-Sod*, *UAS-Sod RNAi* and *He-Gal4>UAS-Sod RNAi*) for 48 h following *Ecc*15 infection (G). Data represent mean ± SD (n = 3). Statistical significance was ascribed as *p<0.05; **p<0.01 and ***p<0.001 as compared to control and **^$^** *p*<0.05; **^$$^** *p*<0.01 and **^$$$^** *p*<0.001 in comparison to respective *He-Gal4*. Scale bar: 20 µm.

RETRACTED

## Discussion

The present study explored the potential of a widely used environmental chemical, Cr(VI), to alter cellular innate immune response using a *Drosophila* model. Cellular immunity of *Drosophila* comprises hemocytes [41], therefore, the observed reduction in total hemocyte count in Cr(VI) exposed *Drosophila* indicates adverse impact of Cr(VI) on cellular immunity. This is corroboration with earlier studies on different model organisms [13], [42]. The altered hemocyte population in exposed *Drosophila* was found to be consistent with the down-regulation of *hemese*, which is expressed in the hemocytes of *Drosophila* larvae [43], in Cr(VI) exposed organism. In addition, phagocytosis has been considered as one of the functional criterions which find significance in order to assess the immunological impact of environmental chemicals [36], [44] on cellular immune function of exposed organism. Therefore, the observed impairment in the ability of hemocytes isolated from Cr(VI) exposed *Drosophila* to phagocytose GFP-labeled *E. coli* indicated that exposure to Cr(VI) has resulted into functional alteration in the hemocyte-mediated immune function. In this regard, previously it has been demonstrated that heavy metals affected the phagocytic activity of the immune cells *in vitro* [45], [46].

The observed alteration in cellular immune response, therefore, may weaken the immune defense of Cr(VI) exposed organism due to reduced immune function since chemical induced impairment in innate defense mechanism was suggested to alter the resistance of exposed organism against microbial infection [3], [47]. The bacterial strain, *Ecc*15, is a natural pathogen of the organism and is reported to induce global immune response in *Drosophila* by natural infection [48]. Thus, enhanced susceptibility against *Ecc*15 infection confirms the immuno-compromised situation of Cr(VI) exposed *Drosophila* larvae. Thus, reduction in total hemocyte population, decreased expression of *hemese*, impaired phagocytic activity and weakened resistance against bacterial infection confirms Cr(VI) induced alteration in cellular immune defense of exposed organism.

RETRACTED

Since we observed that Cr(VI) affects cellular immune response in exposed organism, the likely reason was explored. In a cellular system, metabolic reduction of Cr(VI) to its lower oxidation states has been reported to generate ROS [9]. The latter has been causally linked to accelerated apoptotic cell death [37]. Therefore, we argued that increased ROS generation in the hemocytes of Cr(VI) exposed *Drosophila* larvae would increase the percent of apoptotic cell population concurrent with significantly increased level of DEVDase activity that eventually may negatively affect the health of hemocytes. The levels of ROS were measured both in terms of O_2_^−^ as well as H_2_O_2_ generation wherein higher level of DHE fluorescence as compared to DCF suggests that Cr(VI) induced generation of O_2_^−^ plays a prominent role in exerting adverse effects of the chemical on *Drosophila* hemocytes. Our observation was supported by a previous *in vitro* study wherein O_2_ **^−^** as the major ROS was shown to be associated with Cr(VI)-induced apoptosis [9]. Besides O_2_ **^−^** as one of the ROS for the observed adverse effects, it is quite likely that other reactive species may influence the above events. Since dismutation of O_2_ **^−^** leads to the formation of H_2_O_2_, we inhibited H_2_O_2_/OH generation in the hemocytes of exposed organism by using an anti-oxidant NAC. However, non-significant change in the total hemocyte count and apoptosis in the hemocytes of NAC and Cr(VI) co-exposed *Drosophila* larvae as compared to Cr(VI)-alone exposed organism suggests that along with O_2_^−^, there is possible involvement of other reactive species instead of H_2_O_2_ in Cr(VI) induced modulation of the cellular immunity. In this context, Szabo et al [49] stated that the reaction between superoxide (O_2_ **^−^**) and nitric oxide (NO) in a biological system can produce peroxynitrite (ONOO^−^) anion. Increased ONOO^−^ formation as evident by increased DHR fluorescence in the hemocytes of Cr(VI) exposed *Drosophila* could likely be the reason for free radical induced cellular injury which was also reported previously in other cell types [49], [50]. Further, to confirm the involvement of ONOO^−^ species in Cr(VI) induced alteration of cellular immune aspects, we inhibited their generation in the hemocytes of *Drosophila* larvae co-exposed to Cr(VI) and L-NAME (NOS inhibitor). Cr(VI) induced adverse effects on hemocytes was shown to be significantly attenuated by L-NAME as compared to Cr(VI)-alone exposed group. To garner support that ONOO^−^ generation is responsible for Cr(VI) induced alterations of cellular immunity in exposed organism, we co-exposed *Drosophila* larvae to SNP (NO generator) and Cr(VI). Deteriorated hemocyte health observed in SNP-Cr(VI) co-exposed organism strengthens the possibility of ONOO**^−^** mediated injury to the hemocytes of Cr(VI) exposed organism.

RETRACTED

Due to generation of reactive species in the hemocytes of Cr(VI) exposed *Drosophila* larvae, status of anti-oxidant defense system in these cells assume biological significance. In this context, significant reduction in SOD activity in the hemocytes of exposed organism suggests that SOD plays a major role as an anti-oxidant enzyme. SOD catalyses the dismutation of O_2_^.−^ radical to O_2_ and H_2_O_2_ [15] and hence decreased enzyme activity further enhances the generation of O_2_^.−^ in the hemocytes of Cr(VI) exposed organism. An increase in O_2_^.−^ generation due to decreased SOD activity supports the formation of ONOO**^−^** because of the favoured reaction between O_2_^.**−**^ and NO in the hemocytes of Cr(VI) exposed organism. Moreover, lower level of H_2_O_2_ formation in the hemocytes of Cr(VI) exposed organism supports our observation of decreased activity of SOD. Interestingly, we observed an increase in DCF fluorescence in the hemocytes of exposed organism in contrast to the observed decrease in CAT activity, which is reported to breakdown H_2_O_2_ to H_2_O and molecular oxygen [51], that is probably due to the sensitivity of DCF against both H_2_O_2_ and ONOO^−^ [52]. Hence, decreased SOD activity along with increased O_2_^.−^ generation in the hemocytes of exposed organism enhances the adversities caused by Cr(VI). In addition, decreased SOD activity in the hemocytes of exposed organism might be due to ONOO**^−^** mediated nitration of SOD which may also reduce the enzyme activity. An increased SOD activity in the hemocytes of Cr(VI) exposed organism following inhibition of ONOO^−^ generation further confirmed the above (Fig. S6). Along with decreased activities of all the tested anti-oxidant enzymes and increase in lipid peroxidation in the hemocytes of Cr(VI) exposed organism, diminished level of TAC further indicates a deterioration in over-all anti-oxidant defense system vis a vis increased oxidative stress in the hemocytes of exposed organism. Thus, generation of O_2_^.**−**^ at higher concentrations of Cr(VI) could be accounted for the oxidative damage to the hemocytes of exposed organism concomitant with increased cell death leading to the down-regulation of cellular immune response.

Based on our observations of increased generation of O_2_^.**−**^ along with significantly decreased SOD activity in the hemocytes of exposed organism, we hypothesized that over-expression of Cu/Zn SOD in the hemocytes of *Drosophila* larvae would provide protection to these cells from Cr(VI) induced adversities. We, therefore, over-expressed *sod* in the hemocytes of *Drosophila* in a targeted manner using *He-Gal4* driver. Contrary to the suppression of cellular immune response in Cr(VI) exposed Oregon R^+^ and in *He-Gal4* strains, significant improvements evident in the *sod* over-expressed strain (*He-Gal4>UAS-Sod*), suggested *sod* governed underlying mechanism of Cr(VI) induced alteration in cellular immunity. In this context, less ROS generation, decreased oxidative stress, appearance of lesser number of apoptotic cells, decreased DEVDase activity and increased survival against *Ecc*15 pathogenicity was observed in the *sod* over-expressing strain. Enhanced SOD activity in the over-expressing strain would cause dismutation of O_2_^.−^ radicals, the major ROS species, shown to be involved in Cr(VI) induced adversities in the hemocytes and in the process would provide beneficial effect on cellular innate immune response of the organism. Our study finds support from an earlier study by Marikovsky et al [53] which has demonstrated that *sod* can play an important role in adaptive immune response. The observed rescuing effect of *sod* over-expression against Cr(VI) induced oxidative injury to the hemocytes of exposed organism prompted us to further assess a situation when SOD is knocked down genetically from the organism. A previous study showed that *Saccharomyces cerevisiae sod1Δ* deletion strain was remarkably more sensitive to adverse effects of Cr(VI) [54]. In the same context, our observations of increased oxidative stress and apoptotic cell death in Cr(VI) exposed *He-Gal4>UAS-Sod RNAi* strain along with poor resistance displayed by these organisms against bacterial infection validates our hypothesis of protective role of SOD on cellular immune response of exposed *Drosophila*. In parallel, similar levels of metal intake in the hemocytes of exposed organism irrespective of strain difference indicate that the observed pattern is independent of strain variation. In spite of comprehensive demonstration of the protective role of SOD in improving the hemocyte health in Cr(VI) exposed organism, possibilities of other cellular machineries taking up parallel roles in this context cannot be ruled out.

RETRACTED

## Conclusions

This study provides evidences that the mechanism of Cr(VI) induced alteration of *Drosophila* cellular immune response involves O_2_^.−^/ONOO^−^ mediated oxidative stress in the hemocytes of *Drosophila* wherein over-expression of an anti-oxidant gene, *sod*, could ameliorate the Cr(VI) induced adversities by preventing oxidative injury (Fig. 10). Based on the conserved pathways for innate immunity existing in *Drosophila* and mammals including human, the present study enhances the broad understanding of chemical induced alterations on immunity in higher organism. Further, *Drosophila* is recommended as a functional *in vivo* model for testing the impact of environmental chemicals on innate immune response with minimum ethical concern.

**Figure 10:** Schematic representation of Cr(VI)-induced alterations on cellular immunity in *D. melanogaster*. Cr(VI) altered cellular innate immune response through O_2_^.−^/ONOO**^−^** mediated oxidative stress in the hemocytes of exposed organism. The induction of oxidative stress leads to caspase-3 activation vis a vis apoptosis in the hemocytes which results into reduction in total hemocyte population in exposed organism. The altered immunity was manifested by decreased resistance of these organisms against pathogenic *Ecc*15 infection. Cr(VI) induced suppression of cellular immunity was subsequently modulated/rescued by over-expressing *sod* in *Drosophila* hemocytes.

## Supporting Information

Figure S1 **Standardization procedure of sample volume for superoxide dismutase (SOD) activity in** ***Drosophila*** **hemocytes.** The SOD activity was standardized in *Drosophila* hemocytes according to the assay procedures described by McCord [27]. In this assay, SOD activity of a sample was measured as the percent inhibition of reduction in cytochrome C at 550 nm. Volume of the sample required in this assay should produce the amount of inhibition in the 40–60% range. The assay was standardized for *Drosophila* hemocytes by plotting the percentage inhibition against the volume of hemocyte sample (µl). The response curve suggests that 40–60% inhibition was observed by using 30 and 40 µl of hemocyte sample where 40 µl sample provides the maximum inhibition in the desired range. Therefore, this sample volume was used for further experiments to calculate SOD activity.
(TIF)

Figure S2 **Optimization procedure for total anti-oxidant capacity (TAC) by ABTS decolorization assay in** ***Drosophila*** **hemocytes.** ABTS decolorization assay was optimized in the hemocytes of *Drosophila* to calculate total anti-oxidant capacity with respect to the trolox standard. In this assay, the anti-oxidant capacity of a sample was measured as the percentage inhibition of the absorbance of ABTS radical cation (ABTS**^•+^**) at 734 nm. The concentration-response curve for the standard reference data was obtained by plotting the percentage inhibition of ABTS**^•+^** against trolox standard (µM) (A). The assay was then optimized for *Drosophila* hemocytes by plotting the percentage inhibition of ABTS**^•+^** against the volume of hemocyte sample (µl) (B). The dose-response curve suggest that 60-80% inhibition of ABTS^•+^ was observed using 10 µl of hemocyte sample. Therefore, this sample volume was used for further experiments.
(TIF)

Figure S3 **Reduced expression of** ***hemese*** **in Cr(VI) exposed** ***Drosophila*** **larvae.** Relative expression of *hemese* in Oregon R^+^ larvae which were exposed to Cr(VI) for 24 and 48 h by qRT-PCR assay (A). Graph showing relative expression of *hemese* in *He-Gal4*, *UAS-Sod*, *He-Gal4>UAS-Sod*, *UAS-Sod RNAi* and *He-Gal4>UAS-Sod RNAi* larvae exposed to Cr(VI) for 48 h (B). Data represent mean values of three independent experiments (20 larvae in each). All the expression values were normalized to experimental endogenous control *gapdh*. Statistical significance was ascribed as **p<0.01; ***p<0.001 in comparison to control and **^$$^** *p*<0.01; **^$$$^** *p*<0.001 in comparison to respective *He-Gal4*.
(TIF)

Figure S4 **Concentration optimization of NAC, L-NAME and SNP for their exposures to** ***D. melanogaster*** **larvae.** The concentration of N-acetylcysteine (NAC), N-nitro-L-arginine methyl ester (L-NAME) and sodium nitroprusside (SNP) was optimized in the hemocytes of *Drosophila* by DCF or DHR fluorescence by drawing concentration response curve for each chemical. The percent inhibition of DCF fluorescence for NAC and percent inhibition/generation in/of DHR fluorescence for L-NAME and SNP was measured in *Drosophila* hemocytes to calculate the concentration of the above chemicals to be used for exposures to *D. melanogaster* larvae. The dose-response curve of NAC (A) was plotted as normalized percent inhibition in DCF fluorescence as against 20.0 µg/ml of Cr(VI) while the same for L-NAME (B) and SNP (C) were plotted as normalized percent inhibition/generation in/of DHR fluorescence. The concentration of each chemical showing maximum/optimum inhibition in DCF/DHR or generation of DHR fluorescence was used for further experiments.
(TIF)

Figure S5 **Measurement of colony forming units (CFU) in Cr(VI) exposed organisms.** Ten infected larvae were surface-sterilized with 70% ethanol after rinsing them with water. Bacterial persistence was then measured by plating larval homogenate on LB medium after 1 h of infection with *Ecc*15 [48]. The analysis of bacterial count was normalized by logarithmic transformation. Bar graph represents the number of colony-forming units (CFU) per larvae in Cr(VI) exposed Oregon R^+^ (A) and *He-Gal4*, *UAS-Sod*, *He-Gal4>UAS-Sod*, *UAS-Sod RNAi*, *He-Gal4>UAS-Sod RNAi* for 48 h (B) larval strains.
(TIF)

Figure S6 **Determination of SOD activity in the hemocytes of** ***Drosophila*** **larvae co-exposed to Cr(VI) and NAC/L-NAME/SNP.** Graphical representation of SOD activity in the hemocytes of 20.0 µg/ml Cr(VI) exposed Oregon R^+^ larvae along with 10 mg/ml N-acetylcysteine (NAC) or 100 mM N-nitro-L-arginine methyl ester (L-NAME) or 50 µM sodium nitroprusside (SNP) after 24 and 48 h respectively. Significant differences were determined as **p<0.01; ***p<0.001 in comparison to control and **^#^** *p*<0.05; **^##^** *p*<0.01; **^###^** *p*<0.001 as compared to 20.0 µg/ml Cr(VI) exposure.
(TIF)

Table S1 **Chromium level (ng/ml) in the hemocytes of different** ***Drosophila*** **larvae.**
(DOC)

RETRACTED

## References

[1] DepledgeMH, GallowayTS (2005) Healthy animals, healthy ecosystems. Front Ecol Environ 3: 251–258.

[2] GavinIM, GillisB, ArbievaZ, PrabhakarBS (2007) Identification of human cell responses to hexavalent chromium. Environ Mol Mutagen 48: 650–657.1768546210.1002/em.20331

[3] HarfordAJ, O'HalloranK, WrightPF (2005) The effects of in vitro pesticide exposures on the phagocytic function of four native Australian freshwater fish. Aquat Toxicol 75: 330–342.1622990310.1016/j.aquatox.2005.09.005

[4] De GuiseS, BernierJ, LapierreP, DufresneMM, DubreuilP, et al (2000) Immune function of bovine leukocytes after in vitro exposure to selected heavy metals. Am J Vet Res 61: 339–344.1071453010.2460/ajvr.2000.61.339

[5] SokolovaIM, EvansS, HughesFM (2004) Cadmium-induced apoptosis in oyster hemocytes involves disturbance of cellular energy balance but no mitochondrial permeability transition. J Exp Biol 207: 3369–3380.1532621310.1242/jeb.01152

[6] BarcelouxDG (1999) Chromium. J Toxicol 37: 173–194.10.1081/clt-10010241810382554

[7] International Agency for Research on Cancer (1990) Chromium and chromium compounds. In: Chromium, Nickel and welding. IARC Monographs on the evaluation of carcinogenic risk of chemicals to humans. Lyon, France. pp. 49–256.

[8] ShrivastavaR, UpretiRK, SethPK, ChaturvediUC (2002) Effects of chromium on the immune system. FEMS Immunol Med Microbiol 34: 1–7.1220860010.1111/j.1574-695X.2002.tb00596.x

[9] AzadN, IyerAK, ManosroiA, WangL, RojanasakulY (2008) Superoxide-mediated proteasomal degradation of Bcl-2 determines cell susceptibility to Cr(VI)-induced apoptosis. Carcinogenesis 29: 1538–1545.1854456210.1093/carcin/bgn137PMC2516494

[10] BagchiD, BagchiM, StohsSJ (2001) Chromium (VI)-induced oxidative stress, apoptotic cell death and modulation of p53 tumor suppressor gene. Mol Cell Biochem 222: 149–158.11678597

RETRACTED

[11] GeethaS, SinghV, RamMS, IlavazhaganG, BanerjeePK, et al (2005) Immunomodulatory effects of seabuckthorn (Hippophae rhamnoides L.) against chromium (VI) induced immunosuppression. Mol Cell Biochem 278: 101–109.1618009510.1007/s11010-005-7095-9

[12] GlaserU, HochrainerD, KloppelH, KuhnenH (1985) Low level chromium (VI) inhalation effects on alveolar macrophages and immune functions in Wistar rats. Arch Toxicol 57: 250–256.387916610.1007/BF00324787

[13] SteinhagenD, HelmusT, MaurerS, MichaelRD, LeiboldW, et al (2004) Effect of hexavalent carcinogenic chromium on carp Cyprinus carpio immune cells. Dis Aquat Organ 62: 155–161.1564884210.3354/dao062155

[14] SugiyamaM (1992) Role of physiological antioxidants in chromium(VI)-induced cellular injury. Free Radic Biol Med 12: 397–407.159227410.1016/0891-5849(92)90089-y

[15] SetoNO, HayashiS, TenerGM (1990) Overexpression of Cu-Zn superoxide dismutase in Drosophila does not affect life-span. Proc Natl Acad Sci U S A 87: 4270–4274.211225010.1073/pnas.87.11.4270PMC54090

[16] HoffmannJA (2003) The immune response of Drosophila. Nature 426: 33–38.1460330910.1038/nature02021

[17] LemaitreB, HoffmannJ (2007) The host defense of Drosophila melanogaster. Annu Rev Immunol 25: 697–743.1720168010.1146/annurev.immunol.25.022106.141615

[18] TirouvanziamR, DavidsonCJ, LipsickJS, HerzenbergLA (2004) Fluorescence-activated cell sorting (FACS) of Drosophila hemocytes reveals important functional similarities to mammalian leukocytes. Proc Natl Acad Sci U S A 101: 2912–2917.1497624710.1073/pnas.0308734101PMC365719

[19] BenfordDJ, HanleyBA, BottrillK, OehlschlagerS, BallsM, et al (2000) Biomarkers as predictive tools in toxicity testing. Altern Lab Anim 28: 119–131.

[20] SinghM, MishraM, SharmaA, ShuklaAK, MudiamMK, et al (2011) Genotoxicity and apoptosis in Drosophila melanogaster exposed to benzene, toluene and xylene: attenuation by quercetin and curcumin. Toxicol Appl Pharmacol 253: 14–30.2142042310.1016/j.taap.2011.03.006

[21] SharmaP, BihariV, AgarwalSK, VermaV, KesavachandranCN, et al (2012) Groundwater contaminated with hexavalent chromium [Cr (VI)]: a health survey and clinical examination of community inhabitants (Kanpur, India). PloS one 7: e47877.2311286310.1371/journal.pone.0047877PMC3480439

[22] AravindhanR, MadhanB, RaoJR, NairBU, RamasamiT (2004) Bioaccumulation of chromium from tannery wastewater: an approach for chrome recovery and reuse. Environ Sci Technol 38: 300–306.1474075110.1021/es034427s

[23] MishraM, SharmaA, ShuklaAK, PragyaP, MurthyRC, et al (2013) Transcriptomic analysis provides insights on hexavalent chromium induced DNA double strand breaks and their possible repair in midgut cells of Drosophila melanogaster larvae. Mutat Res 747–748: 28–39.10.1016/j.mrfmmm.2013.04.00523628323

RETRACTED

[24] MarcuO, LeraMP, SanchezME, LevicE, HigginsLA, et al (2011) Innate immune responses of Drosophila melanogaster are altered by spaceflight. PloS one 6: e15361.2126429710.1371/journal.pone.0015361PMC3019151

[25] WangX, MandalAK, SaitoH, PulliamJF, LeeEY, et al (2012) Arsenic and chromium in drinking water promote tumorigenesis in a mouse colitis-associated colorectal cancer model and the potential mechanism is ROS-mediated Wnt/beta-catenin signaling pathway. Toxicol Appl Pharmacol 262: 11–21.2255236710.1016/j.taap.2012.04.014PMC4429765

[26] LimSY, JangJH, NaHK, LuSC, RahmanI, et al (2004) 15-Deoxy-Delta12,14-prostaglandin J(2) protects against nitrosative PC12 cell death through up-regulation of intracellular glutathione synthesis. J Biol Chem 279: 46263–46270.1531943310.1074/jbc.M406555200

[27] McCord JM (1999) Analysis of superoxide dismutase activity. Curr Protoc Toxicol Chapter 7 Unit 737.3.1–7.3.9.10.1002/0471140856.tx0703s0023045062

[28] SinhaAK (1972) Colorimetric assay of catalase. Anal Biochem 47: 389–394.455649010.1016/0003-2697(72)90132-7

[29] KanzokSM, FechnerA, BauerH, UlschmidJK, MullerHM, et al (2001) Substitution of the thioredoxin system for glutathione reductase in Drosophila melanogaster. Science 291: 643–646.1115867510.1126/science.291.5504.643

[30] MissirlisF, UlschmidJK, Hirosawa-TakamoriM, GronkeS, SchaferU, et al (2002) Mitochondrial and cytoplasmic thioredoxin reductase variants encoded by a single Drosophila gene are both essential for viability. J Biol Chem 277: 11521–11526.1179672910.1074/jbc.M111692200

[31] OhkawaH, OhishiN, YagiK (1979) Assay for lipid peroxides in animal tissues by thiobarbituric acid reaction. Anal Biochem 95: 351–358.3681010.1016/0003-2697(79)90738-3

[32] LowryOH, RosebroughNJ, FarrAL, RandallRJ (1951) Protein measurement with the Folin phenol reagent. J Biol Chem 193: 265–275.14907713

[33] ReR, PellegriniN, ProteggenteA, PannalaA, YangM, et al (1999) Antioxidant activity applying an improved ABTS radical cation decolorization assay. Free Radic Biol Med 26: 1231–1237.1038119410.1016/s0891-5849(98)00315-3

[34] WeydertCJ, CullenJJ (2010) Measurement of superoxide dismutase, catalase and glutathione peroxidase in cultured cells and tissue. Nat Protoc 5: 51–66.2005738110.1038/nprot.2009.197PMC2830880

[35] BassetA, TzouP, LemaitreB, BoccardF (2003) A single gene that promotes interaction of a phytopathogenic bacterium with its insect vector, Drosophila melanogaster. EMBO Rep 4: 205–209.1261261310.1038/sj.embor.embor730PMC1315828

[36] FournierM, CyrD, BlakleyB, BoermansH, BrousseauP (2000) Phagocytosis as a Biomarker of Immunotoxicity in Wildlife Species Exposed to Environmental Xenobiotics. Amer Zool 40: 412–420.

RETRACTED

[37] SonYO, HitronJA, WangX, ChangQ, PanJ, et al (2010) Cr(VI) induces mitochondrial-mediated and caspase-dependent apoptosis through reactive oxygen species-mediated p53 activation in JB6 Cl41 cells. Toxicol Appl Pharmacol 245: 226–235.2029870910.1016/j.taap.2010.03.004PMC5051966

[38] TroyCM, DerossiD, ProchiantzA, GreeneLA, ShelanskiML (1996) Downregulation of Cu/Zn superoxide dismutase leads to cell death via the nitric oxide-peroxynitrite pathway. J Neurosci 16: 253–261.861379110.1523/JNEUROSCI.16-01-00253.1996PMC6578729

[39] ConnersW, WhitebeckC, ChicesterP, LeggetR, LinAD, et al (2006) L-NAME, a nitric oxide synthase inhibitor, diminishes oxidative damage in urinary bladder partial outlet obstruction. Am J Physiol Renal Physiol 290: F357–363.1617486610.1152/ajprenal.00261.2005

[40] LozinskyOV, LushchakOV, StoreyJM, StoreyKB, LushchakVI (2012) Sodium nitroprusside toxicity in Drosophila melanogaster: delayed pupation, reduced adult emergence, and induced oxidative/nitrosative stress in eclosed flies. Arch Insect Biochem Physiol 80: 166–185.2269276810.1002/arch.21033

[41] Evans CJ, Sinenko SA, Mandal L, Martinez-Agosto JA, Hartenstein V, et al.. (2008) Genetic dissection of hematopoeisis using Drosophila as a model system. Advances in Developmental Biology: Elsevier. pp. 259–299.

[42] CiacciC, BarmoC, FabbriR, CanonicoB, GalloG, et al (2011) Immunomodulation in Mytilus galloprovincialis by non-toxic doses of hexavalent Chromium. Fish Shellfish Immunol 31: 1026–1033.2192527310.1016/j.fsi.2011.09.002

[43] KuruczE, ZettervallCJ, SinkaR, VilmosP, PivarcsiA, et al (2003) Hemese, a hemocyte-specific transmembrane protein, affects the cellular immune response in Drosophila. Proc Natl Acad Sci U S A 100: 2622–2627.1259865310.1073/pnas.0436940100PMC151390

[44] GallowayTS, DepledgeMH (2001) Immunotoxicity in invertebrates: measurement and ecotoxicological relevance. Ecotoxicology 10: 5–23.1122781710.1023/a:1008939520263

[45] FugereN, BrousseauP, KrzystyniakK, CoderreD, FournierM (1996) Heavy metal-specific inhibition of phagocytosis and different in vitro sensitivity of heterogeneous coelomocytes from Lumbricus terrestris (Oligochaeta). Toxicology 109: 157–166.865854610.1016/0300-483x(96)03315-x

[46] SauveS, BrousseauP, PellerinJ, MorinY, SenecalL, et al (2002) Phagocytic activity of marine and freshwater bivalves: in vitro exposure of hemocytes to metals (Ag, Cd, Hg and Zn). Aquat Toxicol 58: 189–200.1200787410.1016/s0166-445x(01)00232-6

[47] BernierJ, BrousseauP, KrzystyniakK, TryphonasH, FournierM (1995) Immunotoxicity of heavy metals in relation to Great Lakes. Environ Health Perspect 103: 23–34.10.1289/ehp.95103s923PMC15188188635436

RETRACTED

[48] BassetA, KhushRS, BraunA, GardanL, BoccardF, et al (2000) The phytopathogenic bacteria Erwinia carotovora infects Drosophila and activates an immune response. Proc Natl Acad Sci U S A 97: 3376–3381.1072540510.1073/pnas.070357597PMC16247

[49] SzaboC, IschiropoulosH, RadiR (2007) Peroxynitrite: biochemistry, pathophysiology and development of therapeutics. Nat Rev Drug Discov 6: 662–680.1766795710.1038/nrd2222

[50] PritchardKAJr, AckermanA, KalyanaramanB (2000) Chromium (VI) increases endothelial cell expression of ICAM-1 and decreases nitric oxide activity. J Environ Pathol Toxicol Oncol 19: 251–260.10983891

[51] KirkmanHN, GaetaniGF (2007) Mammalian catalase: a venerable enzyme with new mysteries. Trends Biochem Sci 32: 44–50.1715805010.1016/j.tibs.2006.11.003

[52] CohnCA, SimonSR, SchoonenMA (2008) Comparison of fluorescence-based techniques for the quantification of particle-induced hydroxyl radicals. Part Fibre Toxicol 5: 1–9.1830778710.1186/1743-8977-5-2PMC2289838

[53] MarikovskyM, ZivV, NevoN, Harris-CerrutiC, MahlerO (2003) Cu/Zn superoxide dismutase plays important role in immune response. J Immunol 170: 2993–3001.1262655210.4049/jimmunol.170.6.2993

[54] SumnerER, ShanmuganathanA, SideriTC, WillettsSA, HoughtonJE, et al (2005) Oxidative protein damage causes chromium toxicity in yeast. Microbiology 151: 1939–1948.1594200110.1099/mic.0.27945-0

